# Hydroxysafflor Yellow A (HSYA) Protects Endplate Chondrocytes Against IL-1*β*-Induced Injury Through Promoting Autophagy

**DOI:** 10.1155/2022/6326677

**Published:** 2022-07-04

**Authors:** Zongyu Zhang, Yongfeng Huo, Zhijing Zhou, Peng Zhang, Jun Hu

**Affiliations:** ^1^Department of Orthopedic, Lianyungang Affiliated Hospital of Nanjing University of Chinese Medicine, Lianyungang, Jiangsu 222000, China; ^2^Department of Orthopedic, The First Affiliated Hospital of Kangda College of Nanjing Medical University, Lianyungang, Jiangsu 222004, China

## Abstract

**Background:**

Intervertebral disc degeneration (IDD) refers to intractable pain in patients' waist and legs, which is caused by internal structural disorder and degeneration of intervertebral. This disease severely affects the quality-of-life of people. It has been reported that hydroxysafflor yellow *A* (HSYA), the active ingredient in safflower extract, could inhibit IL-1*β*-induced apoptosis of endplate chondrocytes. However, the mechanism by which HSYA regulates the occurrence and progression of IDD remains unclear.

**Methods:**

Rat endplate chondrocytes were isolated from the intervertebral disc. Next, toluidine blue staining and collagen II immunofluorescence staining were used to identify endplate chondrocytes. Then, MDC staining was used to detect the autophagy of endplate chondrocytes. In addition, Western blot was used to measure the expression of cleaved caspase 3, LC-3I/II and ATG7 in endplate chondrocytes.

**Results:**

IL-1*β* obviously inhibited the viability and proliferation of endplate chondrocytes, while these phenomena were notably reversed by HSYA. Additionally, HSYA was able to inhibit IL-1*β*-induced apoptosis of endplate chondrocytes. Moreover, HSYA protected endplate chondrocytes against IL-1*β*-induced inflammation via inducing autophagy.

**Conclusion:**

HSYA protected rat endplate chondrocytes against IL-1*β*-induced injury via promoting autophagy. Therefore, the present study might provide some theoretical basis for exploring novel and effective methods for patients with IDD.

## 1. Introduction

Intervertebral disc degeneration (IDD) refers to intractable pain in patients' waist and legs which is caused by internal structure disorder and degeneration of intervertebral disc [1, 2]. The main manifestations of IDD including dehydration and herniation of the nucleus pulposus, laceration of the annulus fibrosus, fissure of the cartilage end plate, and ossification of the cartilage end plate [1, 3]. Thus, IDD severely affects the life quality of patients [4, 5]. In recent years, the incidence of IDD has been increasing in younger people [6, 7]. It is report that genetic factors, age, and nutritional status might lead to the occurrence of IDD [8, 9]. At present, the main clinical treatments for IDD are drug therapy and surgery; however, the therapeutic effect of these strategies remains unsatisfactory [5].

Hydroxysafflor yellow *A* (HSYA), a component of safflower, which was reported to exhibit neuroprotective, antioxidant, anti-inflammatory and other pharmacological activities in many diseases [10]. In addition, Yang, Liao reported that HSYA might serve as a potential agent to treat IDD [11]. For example, HSYA could significantly inhibit the apoptosis of endplate chondrocytes during the progression of IDD [11]. However, the mechanism by which HSYA regulates the occurrence and progression of IDD remains unclear.

Autophagy is the process of engulfing cytoplasmic proteins or cellular organelles by cell itself [12]. The process of autophagy is characterized by lysosome formation and the degration of encapsulated contents [13]. As we know, autophagy is able to maintain the metabolic needs of cells and the renewal of some organelles [12, 13]. Moreover, autophagy plays a crucial role in IDD progression [14]. For example, Yurube et al. showed that mTOR complex 1 (mTORC1) protected intervertebral disc cells against inflammatory-induced apoptosis by inducing autophagy [15]. It is well known that mTORC1, the target of rapamycin, could be downregulated by the TSC1/2 (tuberous sclerosis complex 1/2), which negatively regulates the process of autophagy [16]. In addition, Zhang et al. indicated that autophagy is closely related to the development of IDD [17]. Therefore, the present study aimed to explore the mechanism by which HSYA regulates the process of IDD from the perspective of autophagy. We hope this research might provide some theoretical basis for exploring novel and effective methods for patients with IDD.

## 2. Materials and Methods

### 2.1. Isolation and Culture of Endplate Chondrocytes of the Rat Intervertebral Disc

Sprague–Dawley (SD) rats (2 month old) were obtained from Charles River Laboratories (Beijing, China). Firstly, SD rats were sacrificed using CO_2_. After that, the skin of the rat's back was cut open, the lumbar spinal columns were removed en bloc under aseptic conditions, and endplate chondrocytes were collected [18]. Next, endplate chondrocytes were digested with 0.2% trypsin for 20 min. Then, endplate chondrocytes were cultured in a specific medium (Procell, Wuhan, China) with 5% CO_2_ at 37°C. A third generation of chondrocyte was used in the experiments. All animal procedures were approved by the Ethics Committee of Xuzhou Medical University Affiliated Hospital of Lianyungang. The National Institutes of Health Guide for the Care and Use of Laboratory Animals was strictly followed.

### 2.2. Identification of Rat Intervertebral Disc Endplate Chondrocytes

Firstly, endplate chondrocytes were fixed with 4% formaldehyde for 15 min. Next, the cells were rinsed with PBS 3 times and stained with 0.1% toluidine blue for 30 min. In addition, endplate chondrocytes were fixed with 4% formaldehyde for 15 min. Next, the cells were rinsed with PBS 2 times and blocked with 1% BSA for 30 min. Then, cells were incubated with the primary antibody (anti-Collagen II) overnight at 4°C. Subsequently, cells were incubated with a fluorescent secondary antibody. Finally, cells were observed under a fluorescence microscope (Olympus Corporation, Tokyo, Japan).

### 2.3. Reagents

HSYA and 3 MA were obtained from MedChemExpress (St. Louis, MA, USA). In this study, 3 MA was used to inhibit cell autophagy.

### 2.4. Cell Viability Assay

A Cell Counting Kit-8 (CCK8) assay (Dojindo, Kumamoto, Japan) was used to detect the viability of endplate chondrocytes. Endplate chondrocytes (5 × 10^3^ cells per well) were seeded into 96-well plates. Subsequently, cells were treated with IL-1*β* (PeproTech, Rocky Hill, NJ, USA) IL-1*β* + HSYA (10 *μ*M) or IL-1*β* + HSYA (10 *μ*M) for 48 h. After that, cells were incubated with10 *μ*L CCK-8 reagents at a 37°C incubator for another 2 h. Then, the optical density at 450 nm was measured with a microplate reader.

### 2.5. EdU (5-Thynyl-2'-Deoxyuridine) Assay

*In vitro* EdU DNA Proliferation Kit (RiboBio Biology, Guangzhou, China) was used to detect the proliferation of endplate chondrocytes. Endplate chondrocytes (4 × 10^5^ cells/well) were seeded into 24-well plates. Subsequently, cells were incubated with 50 *μ*L PBS containing 4% formaldehyde at room temperature for 30 min. After that, cells were stained with 50 *μ*M EdU (100 *μ*L) for 2 h, and then stained with a fluorescence dye, Apollo567, for 30 min at room temperature in the dark. The nuclei were stained with DAPI (4 *μ*g/ml) for 1 h at room temperature. Finally, cells were observed under a fluorescence microscope.

### 2.6. Flow Cytometry Assay

The annexin V-FITC Apoptosis Detection Kit (Beyotime, Shanghai, China) was used to detect the apoptosis of endplate chondrocytes. Endplate chondrocytes (5 × 10^4^ cells/well) were seeded into 6-well plates. Then, cells were incubated with 5 *μ*L Annexin V-FITC and PI at 4°C in the dark. After that, the apoptosis of endplate chondrocytes was detected by flow cytometry.

### 2.7. Western Blot Assay

All protein was extracted from endplate chondrocytes using RIPA buffer (Aspen Biotechnology, Wuhan, China), and the protein concentration was measured using the BCA protein assay (Aspen). Then, the SDS-PAGE with a volume fraction of 10% was prepared and used to separate protein (40 *μ*g/lane). Electrophoresis (100 V) was stopped when the target protein reached the middle of the gel. Next, protein was transferred onto PVDF membranes and blocked with TBST containing 5% skim milk for 1 h at room temperature. After that, the protein was incubated with primary antibodies (anti-cleaved caspase 3 (ab32042), anti-LC-3I/II (ab128025), anti-ATG7 (ab52472) and anti-*β*-Actin (ab8226)) overnight at 4°C. Subsequently, membranes were incubated with HRP-conjugated secondary antibody (ab7090, 1 : 5000) at room temperature for 1 h. Finally, an enhanced chemiluminescence (ECL) kit (Thermo) was used to observe protein bands. *β*-Actin is used as a loading internal control. All the antibodies were obtained from Abcam (Cambridge, MA, USA).

### 2.8. Immunohistochemical (IHC) Staining

Endplate chondrocytes were fixed in 4% formaldehyde. Later on, the primary antibody (anti-LC-3) was added to the cells at 4°C overnight. After that, cells were incubated with the secondary antibody at room temperature for 1 h. Later on, cells were washed with PBS for 3 times, followed by incubation with 50 *μ*L DAPI solution at room temperature for 5 min. Finally, cells were observed under a fluorescence microscope. All the antibodies were obtained from Abcam.

### 2.9. Monodansylcadaverine (MDC) Staining

The MDC Detection Kit was provided by Jiangsu KeyGEN BioTech (Jiangsu, China). Firstly, endplate chondrocytes were seeded into 24-well plates. Next, 100 *μ*L MDC dyeing solution was added to each well. Then, cells were incubated with MDC dye for 15 min at room temperature. Later on, a fluorescence microscope was performed to observe the stained cells.

### 2.10. ELISA Assay

The expression of IL-6 and TNF-*α* was detected using Rat IL-6 and Rat TNF-*α* ELISA Kits according to the manufacturer's instructions. All these kits were purchased from ELK Biotechnology (Wuhan, Hubei, China).

### 2.11. Reactive Oxygen Species (ROS) Analysis

The production of ROS in endplate chondrocytes was detected using the Reactive Oxygen Species Assay Kit (Beyotime; cat no. S0033S). Endplate chondrocytes were incubated with 2, 7-dichlorofluorescin diacetate (DCFH-DA) for 30 min at 37°C in the darkness. Later on, the cells were collected and subsequently resuspended with PBS. After that, the fluorescence was detected using flow cytometry. DCFH-DA is a fluorescent dye, which is able to detect the activity of hydroxyl, peroxyl, and other ROS in the cell. The principle of the DCFH-DA assay is based on the diffusion of DCFH-DH into the cell. DCFH-DA is first deacetylated by cellular esterases to a nonfluorescent compound (DCFH), which is later oxidized by ROS into DCF. DCF highly express fluorescence and could be detected by fluorescence spectroscopy at 485 nm/535 nm.

### 2.12. Statistical Analysis

Each experiment was repeated at least 3 times. GraphPad Prism software was used to analyze these data. All experimental data was expressed as the mean ± S.D. One-way analysis of variance (ANOVA) and followed by Tukey's tests were used to detect the significance of differences between groups.

## 3. Results

### 3.1. HSYA Reverses IL-1*β*-Induced Growth Inhibition of Endplate Chondrocyte

We first isolated endplate chondrocytes of rat intervertebral disc accordingly to previous report [18]. To identify the isolated rat intervertebral disc endplate chondrocytes, toluidine blue and collagen II immunofluorescence staining were performed. The result of toluidine blue staining indicated the cultured chondrocytes were blue (Figure 1(a)); immunofluorescence staining showed that cultured cells highly expressed collagen II (Figure 1(b)). The above data indicated that the cultured cells were inconsistent with the features of chondrocytes [19]. Next, the effect of HSYA on cell growth was evaluated with the CCK8 assay. The result indicated HSYA inhibited the viability of endplate chondrocytes in a dose-dependent manner (Figure 1(c)). Meanwhile, 10 *μ*M or 25 *μ*M HSYA had very limited cytotoxicity, while 50 *μ*M HSYA significantly inhibited cell viability (Figure 1(c)). Thus, we used 10 *μ*M or 25 *μ*M HSYA in the following experiments.

Additionally, IL-1*β* obviously inhibited the viability and proliferation of endplate chondrocytes. However, these phenomena were notably reversed in the emergency of HSYA (Figures 1(d) and 1(e)). All these data suggest that HSYA notably reversed IL-1*β*-induced growth inhibition of endplate chondrocytes.

### 3.2. HSYA Reverses IL-1*β*-Induced Apoptosis of Endplate Chondrocytes

To investigate the function of HSYA in IL-1*β*-induced endplate chondrocyte apoptosis, flow cytometry was performed. As revealed in Figure 2(a), IL-1*β* markedly induced the apoptosis of endplate chondrocytes, while this phenomenon was reversed by HSYA treatments. Meanwhile, the level of cleaved caspase 3 in endplate chondrocytes was significantly upregulated by IL-1*β*, which was completely reversed by HSYA (Figures 2(b) and 2(c)). To sum up, HSYA could reverse IL-1*β*-induced apoptosis of endplate chondrocytes.

### 3.3. HSYA Induces the Autophagy of Endplate Chondrocytes

It has been reported that LC-3 could promote the formation of autophagosomes, and MDC level reflected the formation of autophagosomes [20, 21]. Thus, LC-3 and MDC staining were performed to investigate the effect of HSYA on cell autophagy. As indicated in Figure 3(a), HSYA significantly increased the level of LC-3 in endplate chondrocytes. In addition, HSYA notably upregulated the level of MDC in endplate chondrocytes (Figure 3(b)). Taken together, HSYA notably induced the autophagy of endplate chondrocytes.

### 3.4. HSYA Induces the Autophagy of IL-1*β*-Treated Endplate Chondrocytes

It is well known that autophagy inhibitor 3 MA is able to inhibit the formation of autophagosomes [22]. To further confirm the function of HSYA on the autophagy of IL-1*β*-treated endplate chondrocytes, 3 MA was used as a negative control. The result of fluorescence staining indicated that IL-1*β* notably upregulated the level of LC-3, and this phenomenon was significantly reinforced by HSYA (Figures 4(a) and 4(b)). As expected, the autophagy promoting effect of HSYA was abolished by 3 MA (Figures 4(a) and 4(b)). Consistently, IL-1*β* significantly enhanced the level of MDC in endplate chondrocytes, and this effect was further enhanced by HSYA (Figure 4(c)). Meanwhile, the promoting effect of HSYA on MDC level was partially reversed by 3 MA (Figure 4(c)).

Additionally, the expression of LC-3 II and ATG7 in endplate chondrocytes was significantly increased by IL-1*β*, and these effects were further enhanced by HSYA (Figure 4(d)). However, the upregulation of LC-3 II and ATG7 was abrogated in the presence of 3 MA (Figure 4(d)). Since ATG7 is known to be the key mediator in cell autophagy [23], it could be suggested that HSYA could promote the autophagy of IL-1*β*-treated endplate chondrocytes.

### 3.5. HSYA Reverses IL-1*β*-Induced Apoptosis in Endplate Chondrocytes by Inducing Autophagy

In order to further explore the mechanism by which HSYA regulated the proliferation of endplate chondrocytes, rescue experiments were performed.

Consistent with the result of Figure 1, HSYA significantly protected endplate chondrocytes against IL-1*β*-induced injury (Figures 5(a) and 5(b)). However, the cell protective effect of HSYA was abolished by 3 MA (Figures 5(a) and 5(b)). In addition, IL-1*β*-induced apoptosis of endplate chondrocytes was notably reserved by HSYA, while 3 MA significantly abolished the effect of HSYA (Figure 5(c)). All these data showed that HSYA was able to reverse IL-1*β*-induced growth inhibition of endplate chondrocyte by inducing autophagy.

### 3.6. HSYA Protects Endplate Chondrocytes Against IL-1*β*-Induced Inflammation Injury

Next, with the purpose of investigating whether HSYA could protect endplate chondrocytes against IL-1*β*-induced inflammation injury, the level of reactive oxygen species (ROS) and inflammatory cytokines was detected. The result indicated that IL-1*β* obviously upregulated the level of ROS in endplate chondrocytes, and this upregulation was reversed by HSYA; however, the effect of HSYA were abolished in the presence of 3 MA (Figures 6(a) and 6(b)). Meanwhile, IL-1*β* significantly increased the expression of IL-6 and TNF-*α* in endplate chondrocytes, while these phenomena were notably reversed in the presence of HSYA (Figures 6(c) and 6(d)). However, the anti-inflammatory effect of HSYA was abolished by 3 MA (Figures 6(c) and 6(d)). In brief, HSYA notably protected endplate chondrocytes against IL-1*β*-induced inflammation injury.

## 4. Discussion

It has been reported that HSYA can significantly reverse the apoptosis of endplate chondrocytes during the progression of IDD [11]. In the current study, HSYA was able to protect endplate chondrocytes against IL-1*β*-induced injury through promoting autophagy. The present study explored the role of autophagy in IL-1*β*-treated endplate chondrocytes; thus, this research might shed new light on exploring new methods against IDD.

The intervertebral disc is a soft tissue structure between two vertebrae that supports and cushions the body [24]. At the same time, the intervertebral disc is the largest nonblood supplying structure of the human body. Therefore, the intervertebral disc easily suffers with aging and degeneration and eventually leads to disc herniation [25]. During the development of IDD, many factors such as inflammation and oxidative stress, may lead to the occurrence of apoptosis and autophagy of endplate chondrocytes [15, 26, 27]. In this study, to establish a cellular model of IDD, IL-1*β* was used to induce chondrocyte injury.

As we know, inflammation and autophagy have a close relationship with the proliferation of chondrocytes [16]. Yang et al. reported that promoting autophagy in articular chondrocytes significantly inhibited inflammation-induced cytotoxicity [16]. Additionally, Ma et al. found BNIP3 notably prevented LPS-induced inflammation and apoptosis of chondrocytes via an increase in autophagy [28]. Consistently, HSYA was able to protect endplate chondrocytes against inflammation via inducing autophagy in the current study. All these data illustrates that autophagy plays a vital role in protecting chondrocytes from inflammation.

More and more studies have shown that traditional Chinese medicine could alleviate the progression of IDD by activating autophagy [29–31]. For example, *β*-Ecdysterone, an important phytosteroid, was able to prevent tert-butyl peroxide-induced apoptosis of nucleus pulposa cells by inducing autophagy [31]. In addition, Yiqi Huoxue recipe inhibited the development of IDD by activating autophagy [29]. Furthermore, resveratrol, a biologically potent natural polyphenol, inhibited oxidative stress-induced disc degeneration by inducing autophagy as well [30]. In the current study, HSYA could attenuate IL-1*β*-induced growth inhibition of endplate chondrocytes via inducing autophagy. The present findings are consistent with previous studies. All these studies commonly suggest that traditional Chinese medicine might serve as a potential and effective agent for the treatment of IDD. Admittedly, the mechanisms by which HSYA inhibits the inflammatory responses in endplate chondrocytes need to be further explored. Thus, more investigations are needed in the coming future.

In conclusion, HSYA protects endplate chondrocytes against IL-1*β*-induced injury through promoting autophagy. Therefore, the present study might provide some theoretical basis for exploring novel and effective methods for patients with IDD.

## Figures and Tables

**Figure 1:** HSYA reverses IL-1*β*-induced growth inhibition of endplate chondrocytes. (a) The chondrocytes were identified using toluidine blue staining. (b) The expression of collagen II was detected by immunofluorescence staining. (c) Endplate chondrocytes were treated with different concentrations (0, 5, 10, 25, 50, or 100 *μ*M) of HSYA. The viability of endplate chondrocytes was detected using CCK-8. (d) Endplate chondrocytes were treated with IL-1*β*, IL-1*β* + 10 *μ*M HSYA, or IL-1*β* + 25 *μ*M HSYA. The viability of endplate chondrocytes was detected using CCK-8. (e) The proliferation of endplate chondrocytes was detected using EdU staining. ^*∗*^*P* < 0.01, ^∗∗^*P* < 0.01 compared with the control group. ^#^*P* < 0.01, ^##^*P* < 0.01 compared with IL-1*β*.

**Figure 2:** HSYA reverses IL-1*β*-induced apoptosis of endplate chondrocytes. (a) Flow cytometry was conducted to detect the apoptosis of endplate chondrocytes. (b and c) The level of cleaved caspase 3 was measured by Western blot. ^∗∗^*P* < 0.01 compared to the control group. ^##^*P* < 0.01 compared to IL-1*β*.

**Figure 3:** HSYA induces the autophagy of endplate chondrocytes. Endplate chondrocytes were treated with 10 *μ*M or 25 *μ*M HSYA. (a) The level of LC-3 in endplate chondrocytes was measured by immunofluorescence staining. (b) MDC staining was used to detect the autophagy of endplate chondrocytes. ^∗∗^*P* < 0.01 compared to control.

**Figure 4:** HSYA induces the autophagy of endplate chondrocytes via mediation of LC-3 and ATG7. Endplate chondrocytes were treated with IL-1*β*, IL-1*β* + 10 *μ*M HSYA, IL-1*β* + 25 *μ*M HSYA, or IL-1*β* + 25 *μ*M HSYA + 3-MA. (a and b) The level of LC-3 in endplate chondrocytes was measured by immunofluorescence staining. (c) MDC staining was used to detect the autophagy of endplate chondrocytes. (d) The level of LC-3 I/II and ATG7 in endplate chondrocytes was tested by Western blot. ^∗∗^*P* < 0.01 compared to the control group. ^##^*P* < 0.01 compared to IL-1*β*. ^^^^*P* < 0.01 compared to IL-1*β* + HAYA (25 *μ*M).

**Figure 5:** HSYA reverses IL-1*β*-induced apoptosis by inducing autophagy. (a) CCK-8 assay was performed to detect the viability of endplate chondrocytes. (b) EdU staining assay was performed to detect the proliferation of endplate chondrocytes. (c) The apoptosis of endplate chondrocytes was detected by flow cytometry. ^∗∗^*P* < 0.01 compared to the control group. ^##^*P* < 0.01 compared to IL-1*β*. ^^^^*P* < 0.01 compared to IL-1*β* + HAYA (25 *μ*M).

**Figure 6:** HSYA protects endplate chondrocytes against IL-1*β*-induced inflammation injury. (a and b) The expression of ROS in endplate chondrocytes was tested by the ROS Assay Kit. (c and d) The expressions of IL-6 and TNF-*α* was measured by ELISA kits. ^∗∗^*P* < 0.01 compared to the control group. ^##^*P* < 0.01 compared to IL-1*β*. ^^^^*P* < 0.01 compared to IL-1*β* + HAYA (25 *μ*M).

## Data Availability

The datasets used and/or analyzed during the current study are available from the corresponding author on reasonable request.
